The article "The Regulatory Effects of MicroRNAs on Tumor Immunity" was published in 2022. Journal: Biomed Res Int.

# The Regulatory Effects of MicroRNAs on Tumor Immunity

**DOI:** 10.1155/2022/2121993

**Published:** 2022-07-20

**Authors:** Yan Lu, Muwen Deng, Kang Wang, Yuanhong Peng, Manzhao Ouyang

**Affiliations:** ^1^GCP Center, Shunde Hospital, Southern Medical University (The First People's Hospital of Shunde Foshan), Foshan 528300, Guangdong, China; ^2^Department of Gastrointestinal Surgery, Shunde Hospital, Southern Medical University (The First People's Hospital of Shunde Foshan), Shunde, Foshan, Guangdong Province 528300, China; ^3^The Second School of Clinical Medicine, Southern Medical University, Guangzhou, Guangdong Province 510080, China

## Abstract

MicroRNAs are endogenous noncoding small RNAs that posttranscriptionally regulate the expressions of their target genes. Accumulating research shows that miRNAs are crucial regulators of immune cell growth and antitumor immune response. Studies on miRNAs and tumors primarily focus on the tumor itself. At the same time, relatively few studies on the indirect regulatory effects of miRNAs in the development of tumors are achieved by affecting the immune system of tumor hosts and altering their immune responses. This review discusses the influence of miRNAs on the antitumor immune system.

## 1. Introduction

For a long time, DNA carrying the information and functional proteins in the functioning of living things had been the research hot spot in gene epigenetic regulation. Scientific studies show that only a small portion of genes in the genomes of humans and other advanced eukaryotes encode for proteins; over 97% of the transcriptional products are from non-protein-coding RNAs. These noncoding RNAs were critical in cell growth, proliferation, differentiation, and apoptosis. Lin-4 is the first miRNA identified that could regulate the developmental timing of C. elegans by acting on the mRNA of the crucial developmental protein lin-14 [1, 2]. Additionally, miRNA let-7 was also found to contribute to the development of C. elegans [3]. miRNAs are small noncoding RNAs or ncRNAs, consisting of a small number of nucleotides, usually 21~23 nt in length. miRNAs regulate gene expression at the posttranscriptional or translational levels by acting in a sequence-specific way, that is, on the 3′-untranslated region (3′-UTR) of the target mRNAs [4, 5]. Furthermore, miRNAs have also been involved in gene silencing (protein degradation factors, such as exosomes) at the pretranslational stage (during chromatin remodeling) and even in the cotranslational stage. Briefly, miRNAs are generated in the nucleus by RNA polymerase II from longer primary transcripts (pri-miRNAs). Pri-miRNAs are usually derived from their introns of protein-coding genes or noncoding genes. Pri-miRNAs fold into hairpins, further bound by Drosha and Dicer, two enzymes from the RNase III family. A microprocessor complex is formed when Drosha interacts with DGCR8 in the nucleus and releases the ~70 nt precursor miRNA (pre-miRNA) hairpin. Following its export to the cytoplasm by exportin-5, Dicer further processes the transcript in order to generate mature ∼20 bp miRNA/miRNA duplexes (Figure 1) [6]. In previous studies, miRNAs accounted for about 1% of the human genome. The miRNA families are critical gene families essential to almost every pathological and physiological process in the body. They are critical in the developmental processes of immune cells. At the same time, they also affect the development of tumors by regulating the immune responses [7, 8].

## 2. miRNAs and Tumor Immunity

### 2.1. miRNAs and Innate Immunity

The innate immune system is the natural immune system, which is gradually formed by organisms during the long-term germline evolution and includes innate immune molecules, innate immune cells (dendritic cells, granulocytes, NK cells, and macrophages), and innate immune barrier. Innate immune molecules and immune cells can rapidly and effectively phagocytose and kill pathogens or “nonself” antigenic foreign bodies in the body. They can recognize antigenic foreign bodies, including pathogens and their products, aging-related injuries, and malformed cells in the body. Nevertheless, cross-reactions can occur if their epitopes are similar enough to those of the original antigen. However, cells in the innate immune system play the dual role of promoting and inhibiting tumor proliferation depending on the surrounding environment [9]. Herein, we mainly focus on the immune cells, including macrophages and dendritic cells (Figure 1).

#### 2.1.1. miRNAs and Macrophages

Depending on their functionally polarized mechanism, macrophages within the tumor microenvironment can either promote or suppress tumor growth. Several miRNAs influence macrophage polarization, which is vital to the progression of cancer, such as extravasation, intravasation, tumor invasion, and premetastatic site formation [10]. For example, miR-21 deficiency induces macrophage polarization to the M1 phenotype in tumor cell environments via the activator of the transcription 1 (STAT1) signaling and the IFN-*γ*/signaling transducer. By downregulating miR-21, STAT1 signaling can be augmented as well as the expression of programmed death-ligand 1 (PD-L1) in macrophages, which inhibits macrophage antitumor activities [11, 12]. Moreover, miR-127 also enhanced macrophage activation, suppressing the expression of M1 marker genes and promoting the transcription of M2 markers [13]. Induction of elevated miR-127 by LPS decreases the expression of BCL6, which inhibits the expression of the phosphatase Dusp1. By reducing Dusp1, the phosphorylation of JNK is increased, which promotes inflammation and the M1 phenotype [13]. In addition, miRNAs can also affect the M2 polarization of macrophages. Veremeyko et al. [14] observed that IL-13 and IL-4 treatment increased the expression of miR-124 and knockdown of miR-124 activated M1 marker expression (i.e., CD86, TNF, and iNOS) while suppressing M2 markers (i.e., Ym1 and CD206) in M2-polarized macrophages [14]. By modulating macrophage polarization, miRNAs have therapeutic potential for treating inflammation-related diseases (Figure 2).

Recent studies have shown that miRNAs regulate macrophage growth, mainly when they interact with macrophage precursors, including hematopoietic stem cells (HSCs), thereby regulating macrophage response to cancer. miR-125a can regulate the survival and implantation of HSCs by silencing proapoptotic factors, such as the BCL2 killing factor (BAK1) and BCL2 modifying factor (BMF) and Krueppel-like factor (KLF) 13 [15]. miRNA-126 expressed in HSCs inhibits cell cycle progression and hematopoietic output through the phosphatidylinositol three-kinase (PI3K)/AKT pathway regulation [16]. Therefore, miRNAs can indirectly affect the growth and development of macrophages through HSCs and by regulating immune-related responses (Table 1).

#### 2.1.2. miRNAs and NK Cells

miRNAs can directly regulate the proliferation and cell lethality in NK cells, along with the regulation of their physiological functions through the introduction of other proteins. NK cells kill the activating receptors as they recognize the non-MHC class I molecule ligands, which in turn affirm the high expression of receptors on the surface of tumors and cells that are infected with viruses while having low expression in normal cells, thereby achieving the targeted goal of killing tumor cells without damaging the normal cells [17]. After overexpression of miR-152, Zhu et al. found that NK cell-mediated cytolysis increased by RT-PCR and WB. The result suggests that miR-152 may act as an immune promoter by upregulating host-mediated cytolysis in NK cells [18]. NK cells and T cells are inhibited by B7-H3, an immunomodulatory glycoprotein on the surface of cells [19]. Although the transcription of B7-H3 is ubiquitous in normal tissues, its protein is preferentially expressed in solid tumor cells only. Xu [20] used PCR to demonstrate that miR-29 levels are high in normal tissues while miR-29 levels are lower in tumors, including brain tumors and sarcomas. Transfection with miR-29 lowers B7-H3 expression, according to the study. The expression of B7-H3 increases after knocking out miR-29, indicating that the transcription of miR-29 is negatively correlated with the expression of B7-H3 [20]. This study was subsequently reported by Asuthkar's team, which further found that the overexpression of miR-29 in MYC+ medulloblastoma cells mediated the downregulation of B7-H3 and inhibited angiogenesis in medulloblastoma. They hypothesized that this biological process might be associated with JAK/STAT1 signaling [21].

#### 2.1.3. miRNAs and Dendritic Cells

miRNAs play the dual role of regulating dendritic cells' (DCs) antigenic transmission and immunogenicity. DCs are professional antigen-presenting cells; immature DCs exhibit strong migration and antigen uptake abilities, whereas mature DCs can modify T cells' viability effectively [22]. Several miRNAs exert positive effects on the immune responses of DCs. Sun et al. show that miR-142 promotes the increase in the inflammatory cytokine production and enhances the T cell activation [22]. miR155 is essential in promoting DC maturation and migration; it can induce the DCs to activate T cells by secreting effector factors. In the breast cancer tumor microenvironment, miR-155 expression in DCs is downregulated, thereby inhibiting the DC-mediated immune response [23]. miRNAs can promote DC-mediated immune reactions and suppress DC-mediated antitumor immune reactions. For instance, miR-21 and miR-28 inhibit the activation and maturation of DCs as well as the activation of T cell-mediated immune reactions [24]. Thus, miRNAs have dual effects on immune responses in DCs.

### 2.2. miRNAs and Adaptive Immunity (Table 1)

Adaptive immunity refers to the immune responses that can be recognized and initiated against a specific pathogen after prior contact with this pathogen [25]. The immune system triggers the immune responses through the lymphocyte-mediated recognition of the corresponding specific antigens and their antigenic receptors by the major histocompatibility complexes (MHCs) involved in several immune cells and immune molecules [26]. The signaling pathways associated with T and B cells are important in specific immunity [27].

#### 2.2.1. miRNAs and Cellular Immunity

The specific immune reactions mediated by T cells are critical to antitumor immunity. Cytotoxic T lymphocytes (CTLs) are the central effector cells in antitumor responses, as they specifically kill mutant cells or tumor cells through the granzyme/perforin pathway and death receptor pathway (TNF-TNFR and Fas-Fasl pathways) [28]. CD4+ Th cells not only activate CD8+ CTLs by releasing several cytokines and enhancing the immune efficacies of CTLs but also produce chemokines, IFNs, and TNF, which directly act on the tumor cells [29].

miRNAs are essential in T cell-mediated tumor immunity. Programmed cell death receptor 1 (PD-1) promotes the apoptosis of antigen-specific T cells in the lymph nodes (programmed cell death) [30]. miRNAs impact T cell exhaustion by regulating PD-1 expression [31]. Li [32] observed increased T cell depletion in melanoma mice. Moreover, miRNA microarray and PD-1 exhaustive analyses showed that the levels of 11 miRNAs changed significantly in the melanoma environment. After screening, it was found that miR-28 could bind to multiple insulin receptor substrates (IRs) and subsequently silence PD-1, thereby attenuating and regulating the depletion of T cells and the expression of PD-1. Zheng et al. [33] also show that miR-155 enhances PD-L1 expression in the diffused sizeable B cell lymphoma microenvironment, wherein CD8+ T cells are recruited by PD-1/PD-L1 interaction, and the function of CD8+ T cells is inhibited by phosphorylated AKT and ERK, in such a way that the efficacy of T cell-mediated tumor immune reactions is reduced.

Additionally, miR-195 and miR-448 also play critical roles in antitumor response pathways. In lung adenocarcinoma, miR-195 acts as a suppressor and regulates the response of CD+4 T cells through the CCDC88C [34]. The T cell is controlled by indoleamine 2,3-dioxygenase (IDO1), which is important to immune tolerance; upregulated expression of IDO1 is reported in several types of cancer [35]. Lou et al. show that IDO1 inhibits the activation of CD8+ T cells in colon cancer. miR-448, a tumor suppressor, attenuates the expression of IDO1 and enhances the activation of CD8+ T cells [36]. The mutual characteristics of miRNAs, PD-1, and other tumor-related molecules have essential value in tumor immunotherapy.

During the development of normal human T cells, they need to undergo gene rearrangement of antigen recognition receptor (TCR), express multiple TCRs, and experience positive and negative selection, which are the core procedures in the growth and development of T cells [37]. miR-181a has a primary function in T cell activation, wherein it regulates thymic selection and the activation threshold of antigen recognition receptors (TCRs) by targeting different signaling pathways [38]. YY1, which modulates TCR signaling by upregulating miR-181a and inhibiting the miR-181a-mediated negative feedback loop, is correlated with a decrease in miR-181a expression. Chu et al. report that insulin receptor 1 (IRS-1), a functional target of miR-126, was increased in the miR-126-knockout mice. The activation, proliferation, and interferon expression of CD4+ T cells were higher than those of the wild-type mice [39]. In conclusion, miRNAs are associated with T cells' activation, development, and maturation.

#### 2.2.2. miRNAs and Humoral Immunity

Multiple genes control B cells during the different stages of development. Previous studies have confirmed that miRNAs are crucial in the growth of normal B cells and the destruction of B cell malignancies; they are expected to provide new markers for clinical diagnosis. It was found that miR-150 has an essential association with c-Myb. miR-150 regulates the differentiation of B cells by targeting c-Myb [40]. In HSCs, there is a high expression of BCR. B cells recognize antigens through BCR, receive antigenic stimulation, and eventually initiate a humoral immune response. Cerna et al. [41] show that DNA damage response (DDR) can activate FOXP1, a positive regulator of BCR; thus, it can be used as an indicator of disease worsening for predicting different clinical courses of chronic lymphocytic leukemia (CCL). Through the DDR/miR-34a axis, B cells can restrict BCR signaling during DDR by downregulating FOXP1. BCR signaling is limited, and antigen delivery and antibody activation are downregulated, indirectly affecting the mechanism of antibody tumor immunity.

## 3. Effects of miRNAs on Tumor Immune Microenvironment

In 1989, the theory of “seed and soil” proposed by Paget explained how tumors survive in their environment; this is the so-called tumor microenvironment (TME) [42]. The tumor microenvironment includes extracellular matrix, tumor cells, peripheral blood vessels, and other nonmalignant cells, along with signaling molecules [43]. Simultaneously, characterized by low oxygen, low pH, high pressure, and nutritional deficiencies, the inhibitory effects of immune molecules and immune cells on the tumor are substantially reduced in the TME; the sensitivity of malignant tumor cells toward chemotherapeutic drugs also reduces significantly [44]. It is becoming increasingly apparent that miRNAs are crucial in the development of tumors by regulating the TME.

Abnormal transduction of signaling pathways in the TME can induce tumor development and enhance the body's immune responses against tumors. In the TME, cancer-associated fibroblasts (CAFs) supply oncogenic signals that support tumor growth, metastasis, and progression. Shen et al. show that miR-206, miR-31, and miR-1can promote the development of lung cancer by regulating FOXO3a/VEGF/CCL2, thereby converting normal fibroblasts into tumor-associated fibroblasts (CAFs) [45].

Exosomes are 20~100 nm small membrane vesicles. After budding from the nucleus, the cell membrane fuses with the small membrane vesicles and then secretes their contents outside the cell [46]. Exosomes contain several functional proteins, mRNAs, and miRNAs [47]. In tumor cells, tumor-derived exosomes (TEXs) are abundantly secreted. They regulate communications between tumor cells and TME, the proliferation of tumor cells, and metastasis of tumor cells [48–50]. Immunosuppressive activity of myeloid-derived suppressor cells (MDSCs) is observed in the TME of immature myeloid cells [51, 52]. MDSCs protect tumor cells from attack by the immune system and thus are tolerant to immunotherapy, posing a significant obstacle to immunotherapy [53]. In recent studies, TEXs have been shown to have essential functions, including activating and expanding MDSCs and suppressing their immune responses [54]. Therefore, TEXs are a vital element of the TME and play a crucial role in tumor development [55]. The miRNA sequencing data from Li et al. show that the expression of miR-21 is high in hypoxic TEXs [56]; the presence of TEXs containing miR-21 in cancer cells can also stimulate MDSCs to suppress the immune system. Existing literature shows that miR-21 overexpression can enhance the amplification and function of MDSCs [57]. Li et al. showed that miR-21 and miR-155 synergistically downregulate the expression of PTEN and SHIP-1, causing t the STAT3 pathway activation, which induced the expansion of MDSCs [57]. Their research provides new evidence for the miR-21-mediated immune escape of MDSCs from the TME. The transmission of anti-VEGFA/CCL2/pre-miR-1, anti-miR-31, and pre-miR-206 inhibits tumor growth, tumor angiogenesis, and lung metastasis when administered systemically [45]. miRs are transported by extracellular vesicles (EVs) and play a critical role in the communication between cells in the TME. Exosomal miRs are involved in reciprocal interaction between the neuroblastoma (NBL) cells and TME components. Thus, it can induce proinflammatory reaction in monocytes and further promote NBL cell chemotherapy resistance [58]. In addition, exosomes from NK and activated NK cells, which contain miRs (mir-186) and cytotoxic proteins (granzymes A and B, granulysin, and perforin), show anticancer activity. By capturing these exosomes, NBL cells inhibit tumor cell growth and migration, preventing tumor cells from escaping from the NK cell-mediated cytotoxic response and inducing apoptosis [59, 60].

## 4. miRNAs and Tumor Immunotherapy

In the last few decades, people have made breakthroughs in understanding how cancer cells escape from the immune system, which in turn has promoted a new insight for preventing the immune escape of tumors. miRNAs have an important impact on tumor development, and similarly, tumor proliferation also counteracts the expression of some miRNA [61, 62].

### 4.1. miRNAs and Immune Checkpoints (ICPs) [63]

As an immunosuppressive pathway, immune checkpoints (ICPs) are critical in maintaining autoimmune tolerance and regulating the duration and range of immune responses in peripheral tissues [64]. miRNAs that regulate the immune system through ICPs are receiving great research attention. ICPs in humans include the B7, the TNF, the CD28, and the TNFR families of proteins, which are popular targets in clinical drug therapy. According to the effect on T cells, ICPs could be classified as cosuppressor proteins (CTLA-4, B7-H4 PD-1, and PD-L1) and costimulatory proteins (ICOS, CD28, B7-H3, B7-H2, CD40, CD40L, CD70, and CD27) [65].

#### 4.1.1. miRNAs and Cosuppressor Proteins

As a member of ICPs, PD-1/PD-L1-related signaling pathways are a research hotspot of tumor immunity due to their effect on the immune escape of cancer cells [66]. Li et al. transfected miR-28 mimics and inhibitors into the B16F10 mouse T cells and evaluated the expression of PD-1 using RT-qPCR. The dual-luciferase report assay of PD-1 3′-UTR indicated that miR-28 could silence PD-1 by combining with PD-1 3′-UTR. At the same time, the miR-28 mimic could also reduce PD-1 expression and silence the 3′-UTR of PD-1 (Table 2) [32]. Wei et al. used RNA22 and miRanda to check whether miR-138 could bind the key ICPs, CLAT-4, and PD-1. After CD4+ T cells were transfected with miR-138, PD-1 and CTLA-4 were downregulated [67]. In a comparative experiment using the glioma mouse model, C57BL/6J, Wei et al. found that the gliomas disappeared gradually in mice transfected with miR-138, while untransfected mice showed continued glioma invasion. Huang et al. transfected the PD-L1 Mut luciferase reporter and PD-L1 WT vectors and miR-374b into T and NK cells; 48 hours after transfection, the PD-L1 WT luciferase activity was significantly lower in the miR-374b group than in the other groups, which confirmed that PD-1 is associated with miR-374b. In the liver cancer model, miR-374b was found to downregulate PD-1 expression and reduce tumor size [68]. miR-374b, miR-138, and miR-28 can aim at the 3′-UTR of PD-L1 mRNA, thereby regulating PD-L1 expression to affect the immunosuppression [64].

CTLA-4 can mediate immunosuppressive pathways and downregulate the activity of T cells [69]. Researchers are trying to enhance the efficacies of tumor vaccines to induce antitumor immune responses by clearing suppressive cells, including Tregs, or blocking immunosuppressive pathways using the CTLA-4 antibodies [70]. Currently, the regulation of the CD28 family by miRNAs remains unclear. By targeting the 3′-UTR of CTLA-4, miR-155 can reduce the production of CTLA-4. At the same time, CD4+ T cell proliferation is significantly enhanced [71]. In miR-155T cell-specific knockout mouse models, ICP blocking treatment against PD-1or CTLA-4 can restore antitumor immune responses [71], which implies that the antibodies of anti-CTLA-4 or anti-PD-1 may be associated with miR-155 overlap. Still, the specific regulatory mechanism needs further investigation.

B7-H4 is expressed chiefly on T cells, B cells, DCs, and macrophages [72]. It is upregulated in colorectal tumor cells [73]. B7-H4 participates in peripheral immune responses and negatively regulates T cell proliferation and immune responses [74]. miRNA-related single-nucleotide polymorphisms (miR-SNPs) are a general term used for a class of functional SNPs that lead to aberrant or lacking miRNA gene regulatory functions [75], which are associated with many complex diseases, including tumors [76]. Wu et al. identified 12 miR-SNPs related to the 3′-UTR of the B7/CD28 family from the NCBI dbSNP BUILED129 and ENSEMBL v58 databases [77]. The constructed related pGL3 vectors of miR-SNPs were cotransfected with the corresponding miRNAs into Chinese hamster ovary cells (CHO cells). miR-1207-5p could significantly inhibit B7-H4 3′-UTR allele expression [77], implying that miR-1207-5p could bond with the 3′-UTR of B7-H4 and inhibit its expression, thereby indirectly regulating the immune response.

#### 4.1.2. miRNAs and Costimulatory Proteins

As T cell-specific molecules, inducible costimulatory molecules (ICOSs) bind specifically to the ligand B7-H2, which leads to ICOS/B7-H2 signaling to stimulate the antitumor response of T cells [78]. T cells in the peripheral blood of tumor patients (such as melanoma and ovarian tumors) express a large amount of ICOSs [79, 80]. ICOS molecules are abundantly expressed in the mouse model tumor treated with anti-CTLA-4 [81], suggesting that ICOS may improve the efficacy of immunotherapy. In a mouse model of colorectal cancer, Wu et al. examined miR-SNPs in the 3′-UTR of the ICOS genes and found that miR-SNPs could substantially weaken the interaction between miRNAs and ICOS, resulting in the upregulation of ICOS expression in T cells [77]. miR-SNPs in ICOS interfere with miR-1279 and miR-2117, inhibit miR-186-5p for ICOS expression, and promote the antitumor responses of T cells. As an immunostimulatory molecule, B7-H2 is primarily expressed in macrophages, DCs, and B cells [82, 83]. It is downregulated in gastric and colorectal cancers [84, 85]. Immune escape of cancer cells in tumors is correlated with B7-H2, but the specific mechanism remains confusing [86]. At present, the only miRNA known to target B7-H2 is miR-24. If the regulatory effect of miR-24 on B7-H2 is disturbed by B7-H2 SNPs, it will increase gastric cancer incidence [87].

### 4.2. miRNAs and CAR-T Cells

Chimeric antigen receptor T cell (CAR-T) is a T cell type having a recombinant receptor against tumor-associated antigens. It combines the affinity of antibodies and the killing activity of T cells, bonds with tumor antigens in an antigen-dependent manner, initiates an activation cascade, and exerts a specific killing effect [88–90]. However, many challenges remain to be addressed in the practical utility of CAR-T therapy as follows [91]: (1) in the treatment using CD19 CAR-T cells, antigen escape frequently occurs, resulting in tumor immune tolerance [92]; (2) CAR-T recognizes healthy tissues and produces nontumor toxicity, which can be life-threatening in severe cases [93]; and (3) due to the complexity of TME of solid tumors, the efficacy of CAR-T is still not promising [94]. Zhang et al. show that miRNA expression levels change in their patient samples after CAR-T treatment. The miRNA-TF (transcription factor) gene network shows that miR-148-3a and miR-375 affect the efficacy of CAT-T by regulating the genes encoding transcription factors and participating in the cross-action CAT-T histone treatment; however, the specific mechanism needs further study [95]. Ohno et al. found that CAT-T cells cotransfected with miR-172-92, as compared to CAT-T without miR-172-92 cotransfection, exhibited better antigenicity in malignant gliomas, which implied that CD19 CAR-T therapy combined with mi-172-92 could improve the problem of antigen escape and enhance the efficacy of CAR-T [96].

Although CD19 CAR-T therapy has entered clinical trials and has been successful in chronic lymphocytic leukemia, its utility is restricted because of the single antibody, rare tumor-specific single antigen, and susceptibility to cross-reactivity, resulting in damage to healthy cells [97]. In 2016, O'Rourke et al. proposed dual-receptor AND-gate T cells. By constructing a T cell circuit that requires the activation of two antigens, only the tumor cells can be targeted and killed by T cells, as they express both antigens simultaneously [98]. Currently, the most commonly used single antigen is CD19CAR-T [99]. Researchers are also studying dual-antigen CAR-T systems such as CD19/CD123 [100] and CD19/CD20 [101]. Immune homeostasis, autoimmunity, and self-antigen regulation are influenced by miRNAs [102]. For example, a lack of miR-146a can deregulate autoantigens and cause autoimmune diseases [103]. The research on the relationship between miRNAs, antigens, and the construction of the double-antigen CAR-T system remains unclear. However, through studies on miRNAs and antigens, the selection of different tumor antigens in double-antigen CAR-T systems, the monitoring of the efficacy of double-antigen CAR-T systems, and the construction of double-antigen CAR-T systems are of utmost significance.

CAR-T cells have made breakthroughs in hematological cancer therapy. However, obstacles remain in CAR-T therapy for solid tumors due to several factors, such as CAR-T cells constrained by the complex microenvironment, diverse immune escape mechanisms, and complex tumor antigen targets in solid tumors. Indoleamine 2,3-dioxygenase 1 (IDO1) may be a target for cancer immunotherapy because it is a standard endogenous mechanism of acquired peripheral immunity. It is an essential indicator for predicting tumor prognosis [104]. In immunodeficient mice, Huang et al. found that miR-153 combined with CAR-T cells effectively improved CAR-T cells' tumor cell killing ability by inhibiting IDO1 [104]. Using CAR-T cells and miRNAs to treat solid tumors opens up an entirely new avenue for immunotherapy. Because of miRNA's oncogenic and tumor suppressor functions, its clinical application has been developed, and relevant novel miRNA drugs have already entered clinical trials. As a phase I clinical trial (NCT02369198^i^) drug, mesomiR-1 delivers miRNA mimics by targeting bacterial minicells. By incorporating miRNA mimics of the tumor suppressor miR-16 in minicells covered with epidermal growth factor receptor (EGFR) antibodies, MesomiR-1 could target tumor cells accurately [105]. In this study, 26 patients with non-small-cell lung cancer (NSCLC) or malignant pleural mesothelioma who tolerated standard treatment were evaluated for the safety of mesomiR-1. The results suggested that mesomiR-1 side effects were within acceptable limits and showed antitumor efficacy in 73% of patients [105]. Thus, this trial provides robust evidence for further studies on the antitumor activity based on miR-16 associated with immune checkpoint inhibitors [106].

## 5. Conclusion

As a class of highly conserved noncoding small RNAs, miRNAs are important in regulating human tumor immunity, including tumor development, progression, invasion, metastasis and antigen presentation, immune-related molecules, and inhibition of cell activation of the entire immune response process (Table 2 and Figure 3). Previous studies on miRNAs and tumors have investigated the relationship between high or low expressions of miRNAs and tumor proliferation and metastasis or the downstream pathways regulated by miRNAs that affect tumor growth. Research has recently shifted to miRNAs and tumor-related immune responses, wherein miRNAs have been found to modulate tumor immune responses. These include the activation of antigen receptor signaling (miR-181a [38]), antigen-presenting cells (miR-28 [32]), cellular differentiation (miR-124 [14] and miR-21 [11]), and immune escape (miR-21 [24]) or immune surveillance (miR-186 [59]). miRNAs are essential in rapidly developing cancer immunotherapy and have good application prospects. miRNAs serve as biomarkers for tumor diagnosis, treatment, and prognosis and critical targets for tumor immunotherapy. This feature may provide a much-warranted breakthrough for tumor immunotherapy and widen its prospects for treating more malignant tumor types, thereby benefitting more patients.

## Figures and Tables

**Figure 1:** miRNA biogenesis.

**Figure 2:** miRNA affects the polarization of macrophages.

**Figure 3:** miRNAs participate in the immune responses.

**Table 1:** The function of miRNAs in adaptive immunity.

miRNA	Type of immunity	Functions	References
miR-28	Cellular immunity	Silences PD-1 and attenuates the exhaustion of T cells	[32]
miR-155	Cellular immunity	Activates the expression of PD-L1	[33]
miR-195	Cellular immunity	Inhibits CD4T cells through CCDC88C	[34]
miR-448	Cellular immunity	Inhibits IDO1 and enhances CD8+ T cell response	[36]
miR-181a	Cellular immunity	Control TCR signal	[38]
miR-126	Cellular immunity	Acts on IRS-1, regulates T cell activation	[39]
miR-150	Humoral immunity	Acts on BCR, controls B cell differentiation	[40]
miR-34a	Humoral immunity	Affects BCR signaling by the DDR/miR-34a axis	[41]

**Table 2:** Cell types and corresponding functions in the main miRNA interactions.

miRNA	Cell types	Functions	References
miR-21	Macrophages	Changes in the polarity of macrophages	[11]
miR-125a	HSCs	Regulates the survival of HSCs	[15]
miR-126	HSCs	Inhibits the cell cycle	[16]
miR-127	Macrophages	Changes in the polarity of macrophages	[13]
miR-124	Macrophages	Promotes the differentiation of M1 macrophages	[14]
miR-152	NK cell	Upregulates the activity of NK cells	[8]
miR-29	NK cell	Regulates NK cells indirectly through B7-H3	[19]
miR-142	DC	Enhances the activation of inflammatory factors	[22]
miR-155	DC	Suppresses DC-mediated immune response	[23]
miR-28	T cell	3′-UTR binds directly to PD-1	[32]
miR-195	T cell	Regulates CD+4 T cell activation by CCDC88C	[34]
miR-448	T cell	Inhibits IDO1	[36]
miR-181a	T cell	Control TCR signal	[38]
miR-126	T cell	Acts on IRS-1, regulates T cell activation	[39]
miR-150	B cell	Acts on BCR, controls B cell differentiation	[40]
miR-1	CAF	Regulates FOXO3a/VEGF/CCL2	[45]
miR-206	CAF	Regulates FOXO3a/VEGF/CCL2	[45]
miR-31	CAF	Regulates FOXO3a/VEGF/CCL2	[45]
miR-186	NK cell	Suppresses immune escape	[59]
miR-142-5p	T cell	Overexpression inhibits the PD-1/PD-L1 pathway	[107]
miR-21	MDSC	Activates MDSC amplification	[57]
miR-138	T cell	Inhibits the expression of CTLA-4 and PD-1	[67]
miR-374b	T cell	Downregulates PD-1	[68]
miR-155	T cell	Inhibits PD-1 and CTLA-4	[71]
miR-1207-5p	CHO cell	Binding to B7-H4 3′-UTR allele	[77]
miR-24	CHO cell	Associated with B7-H2	[87]
miR-172-92	CAR-T cell	Enhances CAR-T cell antigenicity	[96]
miR-153	CAR-T cell	Inhibits IDO1, enhances cell lethality	[104]

## Data Availability

Data sharing is not applicable to this article as no datasets were generated or analyzed during the current study.

## Additional Points

*Resources*. This study is registered with https://clinicaltrials.gov/ct2/show/NCT02369198.
